RETRACTED

# The High Risk Factors and Preventive Measures of Percutaneous Nephrolithotomy under the Guidance of B-Ultrasound in the Treatment of Postoperative Renal Calculi

**DOI:** 10.1155/2022/1287910

**Published:** 2022-07-21

**Authors:** Dongshan Pan, Deshi Hong, Fei Wang, Jiebin Lin, Enming Yang, Shixian Wang, Junlong Wang, Xufeng Huang, Kang Li, Lele Yang, ShuiFa Yang

**Affiliations:** Department of Urology Surgery, The Second Affiliated Hospital of Xiamen Medical College, Xiamen, Fujian 361026, China

## Abstract

**Objective:**

The aim of this study is to explore and analyze the high risk factors and preventive measures of percutaneous nephrolithotomy under the guidance of B-ultrasound in the treatment of postoperative renal calculi.

**Methods:**

The clinical data of 220 patients with renal calculi admitted to our hospital from 2018 to October 2021 were retrospectively analyzed. All patients were treated with percutaneous nephrolithotomy *n* = 36) and nonbleeding group (*n* = 184), comparing the personal data, disease-related data, surgical operation related data of the two groups of patients, single factor and logistic multifactor regression analysis to explore the influence of B-guided percutaneous. Nephrolithotomy is a high-risk factor for postoperative bleeding in patients with kidney stones, and preventive measures are based on high-risk factors.

**Results:**

There was no significant difference in the proportion of patients with different genders, whether they had renal surgery, whether they had hypertension, and those with postoperative hepatic insufficiency in the hemorrhagic group and the nonbleeding group (*p* > 0.05). There was no significant difference in age and body mass index between the bleeding group and the nonbleeding group (*p* > 0.05). The proportion of patients with diabetes in the bleeding group was higher than that in the nonbleeding group, and the difference between the groups was statistically significant (*p* < 0.05). Compared with the nonbleeding group, the bleeding group had a higher proportion of patients with calculus diameter ≥2 cm. The proportion of patients with staghorn calculi in the bleeding group was higher than that in the nonbleeding group. The difference between the groups was statistically significant (*p* < 0.05). There was no significant difference in the proportion of patients with hemorrhage, single or multiple renal stones, and ureteral stones in the hemorrhage group compared with the nonbleeding group (*p* > 0.05). Compared with the nonbleeding group, the proportion of patients with bleeding in the first stage was higher, and the proportion of patients with operation time >90 min was higher. The difference between the groups was statistically significant (*p* < 0.05). There was no significant difference in the proportion of patients in the bleeding group compared with the nonbleeding group (*p* > 0.05). Using Logic multifactorial regression analysis, independent risk factors for bleeding after percutaneous nephrolithotomy under ultrasound-guided bovery include diabetes mellitus, stone diameter, staghorn kidney stones, surgical timing, and staging surgery (*p* < 0.05).

RETRACTED

**Conclusion:**

The independent high-risk factors affecting bleeding after percutaneous nephrolithotomy guided by B-ultrasound include diabetes, stone diameter, staghorn type kidney stones, operation time, and staged surgery. According to this, effective preventive measures can effectively reduce the operation and the occurrence of postbleeding.

## 1. Introduction

Nephrolithiasis is one of urinary system disease with a high incidence in clinical studies. Young people and middle-aged men are susceptible groups. Clinically, low back pain and swelling of different degrees often occur, which are serious enough to affect the quality of life of patients. In recent years, continuous innovations of medical operation technology have led to the effective development of minimally invasive technology. Percutaneous nephrolithotomy (PCNL) has been widely used in surgical operations for kidney stones. Effective and complete removal of stones is beneficial to postoperative rehabilitation [1]. However, in actual research, it is found that some patients are prone to suffer complications after PCNL, in which postoperative bleeding is the most common complication. How to take effective measures to avoid postoperative bleeding is a critical problem, which is faced by many urologists. In this study, we analyzed the high-risk factors affecting postoperative bleeding after PCNL under the guidance of B-ultrasound in our hospital in order to find effective preventive ways for postoperative bleeding.

## 2. Materials and Methods

### 2.1. General Information

The clinical data of 220 patients with nephrolithiasis admitted to our hospital from September 2018 to October 2021 were retrospectively analyzed. This group of patients met the relevant diagnostic criteria in the “Guidelines for the Diagnosis and Treatment of Urological Diseases in China (2014 Edition)” [2]. The diagnosis was made after B-ultrasound, urinary tract film, or renal CT examination, and the location, size, and shape of kidney stones were judged. Routine examination showed that the body's blood and urine routine, the heart, brain, liver, and kidney functions were in line with the standard of surgical treatment. Exclude severe cardiac insufficiency, those who cannot tolerate surgical anesthesia, those with obvious or potential renal tumors, those with more than 2 signs of urine routine leukocytes, and those with positive urine cultures; all patients signed informed consent for this trial. All patients were treated with percutaneous nephrolithotomy and were divided into bleeding group (*n* = 36) and nonbleeding group (*n* = 184) according to postoperative bleeding.

RETRACTED

## 3. Methods

All patients were treated with B-ultrasound-guided percutaneous nephrolithotomy: after continuous epidural general anesthesia, the lithotomy position was taken, the ureteroscope was placed in the urethra, and the opening of the ureter was explored. Using the monitoring function of the cystoscope, a 6F ureteral catheter was inserted into the affected side. After the operation was completed, the rigid ureteroscope was withdrawn, the 16F catheter was indwelled, the body position was changed, and normal saline was added to the end of the ureteral catheter [3]. Positioning under the guidance of B-ultrasound, select 18G for puncture treatment of the renal calyx and withdraw the puncture needle after the successful insertion of the guide wire. Use a 12F fascia dilator along the guide wire to expand the channel to complete the operation of expelling urine, insert a flexible ureteroscope into it through the scope sheath, observe and determine whether there is a stone, and then use the EMS system to complete the suction and suction of the stone. Stone crushing and other operations followed by conventional irrigation of stone [4].

### 3.1. Observation Indicators

The personal data, disease-related data, and surgical operation-related data of the two groups of patients were compared. Univariate and logistic multivariate regression analysis was used to explore the high-risk factors affecting postoperative bleeding after B-ultrasound-guided percutaneous nephrolithotomy for renal calculi. Develop preventive countermeasures based on high-risk factors. (1) Personal information includes gender, age, body mass index, history of renal surgery, hypertension, diabetes, and liver insufficiency; (2) Disease-related data including stone diameter, degree of hydronephrosis, presence of staghorn stones, single or multiple kidney stones, and ureteral stones; (3) The operation-related information includes staged operation, operation time, and puncture route. Definition of staged surgery: at the same time or when a new channel needs to be established for stage II quariogenesis, puncture dilation and stonemaking extraction are defined as first stage quarry; the extraction of stones through the original channel after the removal of a stage fistula or stone is defined as the second stage of stone extraction [5]. The degree of hydronephrosis is divided into four degrees: mild, moderate, severe, and extremely severe according to the shape of the renal sinus and the changes in the parenchyma of the echo zone.

RETRACTED

### 3.2. Statistical Processing

SPSS18.0 statistical software was used to analyze the data, the enumeration data was analyzed by *χ*^2^ test, and the measurement data was analyzed by *t*-test. *p* < 0.05 represents statistical significance.

## 4. Results

### 4.1. Univariate Analysis of the General Data of the Two Groups

There was no significant difference in the proportion of patients with different genders, history of renal surgery, hypertension, and liver insufficiency between the bleeding group and the nonbleeding group (*p* > 0.05). There was no significant difference in age and body mass index between the bleeding group and the nonbleeding group (*p* > 0.05). Compared with the nonbleeding group, the proportion of diabetic patients in the bleeding group was higher, and the difference between the groups was statistically significant (*p* < 0.05), as shown in Table 1.

### 4.2. Univariate Analysis of Disease-Related Data between the Two Groups

Compared with the nonbleeding group, the proportion of patients with stone diameter ≥ 2 cm in the bleeding group was higher, and the proportion of patients with staghorn stones was higher in the bleeding group than in the nonbleeding group, and the difference between the groups was statistically significant (*p* < 0.05). Compared with the nonbleeding group, the proportion of patients with different degrees of hydronephrosis, single or multiple renal calculi, and ureteral calculi had no significant difference (*p* > 0.05), as shown in Table 2.

### 4.3. Univariate Analysis of Surgical Operation-Related Data between the Two Groups

Compared with the nonbleeding group, the bleeding group had a higher proportion of patients with one-stage lithotripsy, and the proportion of patients with operation time >90 min was higher, and the difference between the groups was statistically significant (*p* < 0.05). There was no significant difference in the proportion of patients under different puncture routes between the bleeding group and the nonbleeding group (*p* > 0.05), as shown in Table 3.

### 4.4. Logistic Multivariate Regression Analysis of High Risk Factors for Postoperative Bleeding after Ultrasound-Guided Percutaneous Nephrolithotomy

Logistic multivariate regression analysis showed that the independent risk factors for bleeding after B-ultrasound-guided percutaneous nephrolithotomy included diabetes, stone diameter, staghorn nephrolithiasis, operation time, and staged operation (*p* < 0.05), as shown in Table 4.

RETRACTED

## 5. Discussion

Stone disease is mainly caused by abnormal mineralization of the human body, usually caused by the accumulation and formation of calcium salts or lipids. Some studies have reported that the occurrence and development of kidney stones are mainly related to the high calcium and protein content in the food eaten. These substances can significantly increase the content of urinary calcium, uric acid, and urinary oxalic acid in the human body, forming an acidic environment, providing an environmental basis for the growth of kidney stones, which has a greater impact on the health of patients [6, 7]. Combined with previous studies, for patients who can tolerate surgery and have poor remission effect of drug therapy, the surgical options include laparoscopic lithotripsy, open lithotripsy, and retrograde ureteroscopic lithotripsy [8, 9]. However, although open lithotripsy can achieve a certain curative effect, there are still obvious defects during the implementation. The more common defects are that the human body is damaged, the amount of intraoperative blood loss is large, and the renal function of patients is also different. Degree of influence and the recovery rate are slow [10, 11]. In recent years, with the continuous development of urological endoscopy technology, B-ultrasound-guided percutaneous nephrolithotomy has made progress and application in the treatment of kidney stones, but the amount of bleeding that may be caused during the operation and the damage to the renal parenchyma has been made [12].

Real-time X-ray guidance is the most commonly used technique for the establishment of percutaneous renal puncture channels, but this method can only show the anatomy of the kidneys, and cannot monitor the position of adjacent organs in real time, increasing the risk of organ damage such as intestinal tubes, liver, and pleural cavity. In addition, real-time X-ray-guided PCNL exposes patients and surgeons to radiation, and although the radiation dose per procedure is low, the risk of exposure to radiation is significantly increased over time. The advantages of PCNL under ultrasound guidance have surpassed with those of PCNL under X-ray perspective guidance. During entry into the pyelonephrenalcup, ultrasound can clearly show the neighboring relationship between the renal structure and surrounding organs, helping clinicians to choose the best puncture path. Percutaneous nephrolithotomy is a common method for the treatment of complicated urinary tract stones in current clinical work. The key point of the operation is to establish a reasonable channel for stone removal and accurately locate the puncture point. The application can better extract the three-dimensional information of the renal collection system and monitor the operation process in real time, ensuring that the operator can identify each operation link in a clear vision. A large number of data show that this type of surgery has the advantages of less trauma to the surrounding tissue, lower complication rate, and faster postoperative recovery compared with the traditional open surgery type [13, 14]. In addition, percutaneous nephrolithotomy is not prone to serious complications in the treatment of kidney stones; especially compared with open surgery, it significantly reduces the amount of intraoperative blood loss, and the safety is guaranteed [15]. However, some clinical research data show that B-ultrasound-guided percutaneous nephrolithotomy is prone to some complications, usually postoperative bleeding, and severe bleeding can lead to the death of patients. Therefore, it is very important to study the independent high-risk factors affecting bleeding after B-ultrasound-guided percutaneous nephrolithotomy in order to formulate effective preventive measures. Combined with the results of this study, it can be seen from the logistic multivariate regression analysis that the independent high-risk factors affecting bleeding after B-ultrasound-guided percutaneous nephrolithotomy include combined with diabetes mellitus, stone diameter, staghorn nephrolithiasis, operation time, and staged surgery (*p* < 0.05).

RETRACTED

The reasons are as follows: (1) The reason why diabetes can cause bleeding after percutaneous nephrolithotomy under the guidance of B-ultrasound is that if the patient is complicated with diabetes, it is easy to cause different degrees of atherosclerosis and microvascular lesions as the disease progresses. It increases the risk of postoperative bleeding. To this end, clinicians need to pay attention to patients with kidney stones combined with diabetes, give hypoglycemic therapy according to the doctor's order, and control the blood sugar level before performing surgical treatment [16]. (2) Although the size of the calculus does not increase the occurrence of postoperative bleeding, the presence of antler stones can easily and significantly increase the number of surgical procedures and require the establishment of multiple channels at the same time. Because the branches of staghorn calculi can extend into one or more calyces, when percutaneous nephroscopy is used, it is easy to cause calyceal neck tear or damage to the renal parenchyma and cause bleeding [17]. For this reason, clinicians need to accurately calculate and analyze the patient's stone volume and other conditions before performing surgical treatment so as to better achieve the purpose of fine operation. (3) When the stone diameter is large, the situation is usually similar to that of staghorn stones, which cannot be treated by single channel, and usually requires multichannel treatment to complete the operation of stone extraction, which increases the damage to the renal parenchyma to a certain extent. In addition, stones with larger diameters cannot be removed at one time and need to be removed after lithotripsy by holmium laser or pneumatic ballistics, which also prolongs the operation time to a certain extent and increases the risk of postoperative bleeding. (4) The results show that the longer the operation time, the greater the impact on the kidney tissue and the higher the risk of bleeding. This requires the operator to make preoperative preparations according to the patient's individual condition and assign clinical work with rich operating experience. The personnel completed the perioperative treatment. (5) In addition, the results of this study found that staged surgery can reduce the occurrence of postoperative bleeding, because the second stage surgery can significantly shorten the operation time of a single operation and greatly reduce the occurrence of operation-related complications. Meanwhile, it can effectively reduce the amount of postoperative bleeding. Therefore, it is recommended that clinicians use staged surgery for patients with poor individual conditions, large stone volume, and long-term lithotripsy to achieve the purpose of reducing postoperative bleeding and safe treatment.

RETRACTED

In summary, the independent high-risk factors affecting bleeding after B-ultrasound-guided percutaneous nephrolithotomy include diabetes mellitus, stone diameter, staghorn nephrolithiasis, operation time, and staged operation. Considering the above risk factors and formulating effective preventive measures will effectively reduce the risk factors and the occurrence of postoperative bleeding.

## Figures and Tables

**Table 1:** Univariate analysis of the general data of the two groups.

High risk factors		Bleeding group (*n* = 36)	Nonbleeding group (*n* = 184)	*χ* ^2^	*p*
Gender	Male	20 (55.56)	86 (46.74)	0.469	0.174
	Female	16 (44.44)	98 (53.26)		

Old (tear)		30.41 ± 2.98	29.78 ± 2.02	0.859	0.135

BMI (kg/m^2^)		25.62 ± 1.75	26.44 ± 1.60	1.136	0.156

Nephrotomyhistory	Yes	4 (11.11)	16 (8.70)	0.106	0.244
	No	32 (88.89)	168 (91.30)		

Combined with hypertension	Yes	8 (22.22)	26 (14.13)	0.754	0.145
	No	28 (77.78)	158 (85.87)		

Combined with diabetes	Yes	32 (88.89)	90 (48.91)	9.739	0.003
	No	4 (11.11)	94 (51.09)		

Combined with hepatic insufficiency	Yes	6 (16.67)	20 (10.87)	0.485	0.165
	No	30 (83.33)	164 (89.13)		

RETRACTED

**Table 2:** Univariate analysis of disease-related data in the two groups.

High risk factors		Bleeding group (*n* = 36)	Nonbleeding group (*n* = 184)	*χ* ^2^	*p*
Renal calculus diameter	<2 cm	6 (16.67)	80 (43.48)	4.454	0.013
	≥2 cm	30 (83.33)	104 (56.52)		

Extent of hydronephrosis	None or mild	20 (55.56)	96 (52.17)	0.069	0.313
	Moderate to severe	16 (44.44)	88 (47.83)		

Staghorn shaped renal calculus	Yes	32 (88.89)	78 (42.39)	13.019	0.0031
	No	4 (11.11)	106 (57.61)		

Renal calculus	Solitary	18 (50.00)	76 (41.30)	0.465	0.177
	Multiple	18 (50.00)	108 (58.70)		

Combined with ureteral calculi	Yes	10 (27.78)	62 (33.70)	0.240	0.283
	No	26 (72.22)	122 (66.30)		

**Table 3:** Univariate analysis of the data related to surgical operations in the two groups.

High risk factors		Bleeding group (*n* = 36)	Nonbleeding group (*n* = 184)	*χ* ^2^	*p*
Staged surgery	Stone extraction at the first phase	26 (72.22)	86 (46.74)	3.912	0.029
	Stone extraction at the second phase	10 (27.78)	98 (53.26)		

Operation time	<60 min	2 (5.56)	60 (32.61)	11.240	0.012
	60∼90 min	6 (16.67)	58 (31.52)		
	>90 min	28 (77.78)	66 (35.87)		

Puncture path	Upper calyx	14 (38.89)	62 (33.70)	0.353	0.198
	Middle calyx	12 (33.33)	58 (31.52)		
	Lower calyx	10 (27.78)	64 (34.78)		

**Table 4:** Logistic multivariate regression analysis of high risk factors for postoperative bleeding after ultrasound-guided percutaneous nephrolithotomy.

High risk factors	Regression coefficients	Standard error	*P*	OR	95%CI
Combined with diabetes	1.298	0.498	0.021	2.983	1.329∼7.983
Renal calculus diameter	1.038	0.404	0.017	2.481	1.409∼6.986
Staghorn shaped renal calculus	0.883	0.366	0.015	1.987	1.276∼3.891
Operation time	1.094	0.487	0.009	2.109	1.449∼5.984
Staged surgery	1.160	0.546	0.007	3.498	1.103∼9.827

## Data Availability

The data can be obtained from the author upon reasonable request.
